RETRACTED

# Sialic acid-modified solid lipid nanoparticles as vascular endothelium-targeting carriers for ischemia-reperfusion-induced acute renal injury

**DOI:** 10.1080/10717544.2017.1410258

**Published:** 2017-11-30

**Authors:** Jing-Bo Hu, Gui-Ling Song, Di Liu, Shu-Juan Li, Jia-Hui Wu, Xu-Qi Kang, Jing Qi, Fei-Yang Jin, Xiao-Juan Wang, Xiao-Ling Xu, Xiao-Ying Ying, Lian Yu, Jian You, Yong-Zhong Du

**Affiliations:** a Institute of Pharmaceutics, College of Pharmaceutical Sciences, Zhejiang University, Hangzhou, China;; b College of Pharmaceutical Sciences, Jiamusi University, Jiamusi, China;; c College of pharmacy, Zhejiang Pharmaceutical College, Ningbo, China

**Keywords:** Sialic acid, nanoparticles, E-selectin, kidney targeting, ischemia reperfusion, acute kidney injury

## Abstract

In an attempt to improve therapeutic efficacy of dexamethasone (DXM)-loaded solid lipid nanoparticles (NPs) for renal ischemia-reperfusion injury (IRI)-induced acute renal injury (AKI), sialic acid (SA) is used as a ligand to target the inflamed vascular endothelium. DXM-loaded SA-conjugated polyethylene glycol (PEG)ylated NPs (SA-NPs) are prepared via solvent diffusion method and show the good colloidal stability. SA-NPs reduce apoptotic human umbilical vein endothelial cells (HUVECs) via downregulating oxidative stress-induced Bax, upregulating Bcl-xL, and inhibiting Caspase-3 and Caspase-9 activation. Cellular uptake results suggest SA-NPs can be specifically internalized by the inflamed vascular endothelial cells (H_2_O_2_-pretreated HUVECs), and the mechanism is associated with the specific binding between SA and E-selectin receptor expressed on the inflamed vascular endothelial cells. Bio-distribution results further demonstrated the enhanced renal accumulation of DXM is achieved in AKI mice treated with SA-NPs, and its content is 2.70- and 5.88-fold higher than those treated with DXM and NPs at 6 h after intravenous administration, respectively. Pharmacodynamic studies demonstrate SA-NPs effectively ameliorate renal functions in AKI mice, as reflected by improved blood biochemical indexes, histopathological changes, oxidative stress levels and pro-inflammatory cytokines. Moreover, SA-NPs cause little negative effects on lymphocyte count and bone mineral density while DXM leads to severe osteoporosis. It is concluded that SA-NPs provide an efficient and targeted delivery of DXM for ischemia-reperfusion-induced injury-induced AKI, with improved therapeutic outcomes and reduced adverse effects.

## Introduction

Renal ischemia-reperfusion injury (IRI) often leads to acute kidney injury (AKI) during kidney transplantation (Aydin et al., 2007), involving complicated pathophysiological mechanisms, including inflammation, apoptosis, and vascular damage. Vascular damage is an initial and important mediator of AKI resulting in the long-term damage and progressive loss of renal function (Basile et al., 2001; Molitoris & Sutton, 2004). Despite advances in clinical and basic studies over the past few decades, therapeutic outcomes of AKI are still poor, with gradually increased morbidity, unavoidable high mortality, and unsatisfactory therapeutic options (Schiffl et al., 2002; Xue et al., 2006). Therefore, treatment of AKI starting from the pathogenesis of the disease to explore a new therapeutic strategy is necessary and crucial.

RETRACTED

E-selectin, a calcium-dependent transmembrane glycoprotein, is dramatically upregulated in in endothelial cells during activated by pro-inflammatory factors, such as tumor necrosis factor-α (TNF-α), interleukin-1 and lipopolysaccharide (LPS) (Van Kampen & Mallard, 2001; Jiang et al., 2015). Once expressed on the surface of cells, it is efficiently internalized by endocytosis (Jubeli et al., 2012). Therefore, E-selectin is a promising target for the site-specific delivery of anti-inflammatory agents. Our previous study has demonstrated that sialic acid (SA)-mediated micelles could be specifically internalized by LPS-activated human umbilical vein endothelial cells (HUVECs) via the specific binding between SA and E-selectin receptor (Hu et al., 2017). Currently, no direct evidence showed whether IRI will lead to the overexpression of E-selectin on vascular endothelial cells. If this hypothesis is feasible, this drug delivery system probably provides a rational basis for exploiting the “vascular targeting’’ strategy to acquire better therapeutic outcomes and avoid drug-induced systemic toxicity for the treatment of renal IRI.

Solid lipid nanoparticles (NPs) are colloidal particles composed of different types of physiological lipids and exhibit a size range between 50 and 400 nm (Hou et al., 2003; Seyfoddin et al., 2010). They are prepared mainly with phospholipids and solid lipids, which are generally considered safe, biocompatible, and biodegradable (Thukral et al., 2014; Misra et al., 2016). They can be a good alternative to polymeric systems due to their unique structure and properties, such as lower toxicity, the ability to protect active pharmaceutical ingredient from chemical degradation, and prolonged drug release. In addition, the possibility to functionalize them with ligands to achieve a site specific targeting makes them more attractive (Pawar et al., 2016; Liu et al., 2017). Therefore, ligand-modified solid lipid NP probably is an ideal delivery system to achieve site-specific and prolonged drug release.

RETRACTED

Dexamethasone (DXM) has been extensively used in the clinical practice for its anti-inflammatory and anti-oxidative stress effects, but several drug-induced systemic toxicities are inevitable. As mentioned above, solid lipid NPs can be used to encapsulate DXM and release preferentially it in inflamed tissues and then reduce its systemic toxicity. To our knowledge, SA-modified solid lipid NPs (SA-NPs) have never been used for the treatment of renal IRI-induced AKI. In this study, DXM-loaded SA-conjugated polyethylene glycol (PEG)ylated NPs (SA-NPs) are prepared for renal IRI-induced AKI. SA-NPs were prepared via solvent diffusion method and its characteristics, including size, polydispersity index, zeta potential, particle morphology, encapsulation efficiency, and loading efficiency, were examined in detail. The target efficacy of SA-NPs was investigated both *in vitro* and *in vivo*. The *in vivo* therapeutic efficacy was assessed in IRI-induced AKI murine models, and evaluation indexes included renal functions, histopathological changes, oxidative stress levels, and pro-inflammatory cytokines. In addition, the specific mechanism of SA-NPs protect vascular endothelial cells from oxidative stress damage was also uncovered.

## Methods

### Materials and animals

DXM and SA were purchased from Aladdin Bio-chem Technology Co. Limited (Shanghai, China). HOOC-PEG-COOH (M_w_ = 2.0 kDa) was purchased from Xi’an ruixi Biological Technology Co., Ltd (Xi’an, China). Fluorescein isothiocyanate (FITC), indocyanine green (ICG), and 3-(4,5-dimethylthiazol-2-yl)-2,5-diphenyltetrazolium bromide (MTT) were purchased from Sigma-Aldrich (St. Louis, MO, USA). A TUNEL assay kit was obtained from Roche (Nutley, NJ, USA). All other solvents were of analytical or chromatographic grade.

ICR mice (body weight: 18 ∼ 20 g) were purposed from the Zhejiang Medical Animal Centre. All animal experiments were carried out in accordance with the National Institutes of Health (NIH, USA) guidelines for the care and use of laboratory animals in research. The surgical procedures and experiment protocols were approved by the Committee for Animal Experiments of Zhejiang University.

### Synthesis and characterization of SA-g-PEG-g-DXM conjugates

SA-g-PEG-g-DXM (SA-PEG-DXM) conjugates were synthesized and the route was provided in Figure S1. Briefly, 2.5 g PEG (1.25 mmol, 1 equiv), 0.775 g Dicyclohexylcarbodiimide (DCC, 3.75 mmol, 3 equiv) and 0.05 g 4-dimethylaminopyridine (DMAP, 0.41 mmol, 0.3 equiv) were added into 20 mL anhydrous dimethyl formamide (DMF), followed by stirring at room temperature for 2 h activate the carboxylic acid of PEG. Then, 0.49 g DXM (1.25 mmol, 1 equiv) was added into this reaction system and stirred for an extra 48 h to produce PEG-DXM. The PEG-DXM was purified by dialysis (MWCO: 3.5 kDa) against deionized water for 2 days, followed by lyophilization.

RETRACTED

The synthesis of SA-PEG-DXM followed the identical protocol as the synthesis of PEG-DXM. Briefly, 1.2 g PEG-DXM (0.5 mmol, 1 equiv), 0.258 g DCC (1.25 mmol, 3 equiv) and 0.016 g DMAP (0.14 mmol, 0.3 equiv) were added into 10 mL anhydrous DMF, then 0.15 g SA was added into the solution and the resulting mixture was stirred for 48 h to produce SA-PEG-DXM. The crude product was purified by dialysis (MWCO: 3.5 kDa) against deionized water for 2 days, followed by lyophilization.

The proton spectra of SA-PEG-DXM were determined using a NMR spectrometer (AC-80, Bruker Bios pin. Germany). Dimethylsulfoxide-*d*_6_ was used as the solvent.

### Preparation and characterization of SA-NPs

SA-NPs were prepared via solvent diffusion method (Yuan et al., 2008). Briefly, weighted SA-PEG-DXM, DXM, glyceryl monostearate (GM, Energy Chemical Co., Ltd, China) and oleic acid (OA, Aladdin Bio-chem Technology Co., Lid, China) were dissolved in 0.5 mL ethanol and rapidly dispersed into 10 mL deionized water under mechanical stirring with 400 rpm at 60 °C for 10 min. After removing ethanol (volatilization at 60 °C), SA-NPs were collected by centrifugation at 20 000 rpm for 15 min, and washed with deionized water to remove unencapsulated DXM and SA-PEG-DXM. In addition, NPs consisting PEG-DXM, DXM, GM, and OA were also prepared in conformity with the identical protocol as the preparation of SA-NPs.

The average diameter, polydispersity index (PDI) and zeta potential of SA-NPs were recorded using dynamic light scattering (Zetasizer, Malvern Co., UK). The SA-NPs solution was diluted to 100 µg/mL with deionized water for measurement. The morphological examination was performed using transmission electron microscopy (TEM, JEOL JEM-1230, Japan), and the samples were overlaid on a formvar-coated copper grid and negatively stained with phosphotungstic acid (2%, w/v) for 1 min.

### Determination of drug entrapment efficiency and drug content

DXM content was determined using high performance liquid chromatograph (HPLC, Agilent 1100, USA) with C18 column (250 mm × 4.6 mm, 5 μm). The mobile phase consisted of methanol and water (v/v = 60:40), and the flow rate was 1.0 mL/min (Xiang et al., 2007). The column temperature and the detection wavelength were set as 25 °C and 240 nm. The entrapment efficiency and drug content were determined via the centrifugal ultrafiltration assay (MWCO: 100 kDa). The SA-NPs solution was centrifuged at 20 000 rpm for 10 min and the unencapsulated DXM and SA-PEG-DXM in filter liquor was determined after dilution with ethanol.

RETRACTED

### *In vitro* release of DXM from SA-NPs

*In vitro* drug release profile of SA-NPs was investigated via the dialysis method (Hazzah et al., 2016), and DXM was determined using HPLC assay. Phosphate buffer (PBS, pH 7.4) was used as dissolution medium.1 mL DXM-loaded SA-NPs was sealed in a dialysis membrane (MWCO: 3500 Da), and then immersed into 40 mL release medium, free DXM and DXM-loaded NPs (equal DXM) as control. This experiment was carried out in an incubator shaker (HZ-8812 S, Taicang, China) maintained at 37 ± 0.5 °C and shaken horizontally at 60 rpm. At predefined time points, the release medium was withdrawn and replaced with fresh medium. The collected DXM was qualified using HPLC assay from the standard DXM curve.

### Cellular uptake of SA-NPs by HUVECs

Fluorescein isothiocyanate isomer I (FITC)-labeled SA-NPs (SA-NPs-FITC) was prepared as following: 1 mg SA-PEG-DXM, 7.7 mg GM, 1 mg OA and 0.3 mg FITC were dissolved in 0.5 mL ethanol and rapidly dispersed into 10 mL deionized water under mechanical stirring with 400 rpm at 60 °C for 10 min. Then, SA-NPs-FITC was collected by centrifugation at 20 000 rpm for 15 min, and subjected to further use. The preparation of NPs-FITC followed the identical procedures as SA-NPs-FITC.

HUVECs were seeded into 24-well Lab-Tek II chamber slides at a density of 5 × 10^4^ cells per well, and incubated for 24 h. Cells were pretreated with 200 µmol/L H_2_O_2_ for 4 h and then incubated with SA-NPs-FITC or NPs-FITC at the concentration of 20 µg/mL for 1, 2 and 6 h, respectively. Cells without H_2_O_2_-pretreatment were used as control. After washed with PBS and fixed with 4% paraformaldehyde solution, cells were visualized using a fluorescence microscope (Olympus, Japan). In addition, flow cytometry was also used for quantificational study

Then, the E-selectin-mediated internalization mechanism of SA-NPs by HUVECs was investigated. HUVECs were seeded in a 12-well plate (5 × 10^5^ cells per well) and cultured for 24 hours, and then exposed to H_2_O_2_ (200 µmol/L). After 4 hours, H_2_O_2_-pretreated HUVECs were incubated with SA-NPs-FITC for 2 h at 37 °C, NPs-FITC as control. After washed with PBS and fixed with cold methanol (−20 °C), cells were incubated with E-selectin antibody (1: 200) for 12 h at 4 °C and then incubated with secondary antibody (1: 500) for 2 h at room temperature. The internalization of SA-NPs and expression of E-selectin receptor was visualized using laser scanning confocal microscope (Zeiss LSM 510 META, Carl Zeiss, Germany). The competitive assay was further performed to demonstrate this E-selectin-mediated internalization mechanism of SA-NPs by HUVECs. Intracellular fluorescence intensity was determined by flow cytometry (FC 500 MCL; Beckman Coulter, USA) during HUVECs with various concentrations of SA (0.5, 1 and 2 mg/mL) at 2 h post-exposure to SA-NPs-FITC.

RETRACTED

### Cell viability

To investigate whether SA-NPs protect HUVECs from oxidative stress damage, a 3-(4,5-dimethylthiazol-2-yl)-2,5-diphenyltetrazolium bromide (MTT) assay was used to assess cell survival (Guo et al., 2012). Briefly, HUVECs were seeded into 96-well plates at a density of 5 × 10^3^ cells per well, and incubated for 24 h. Then, cells pretreated with H_2_O_2_ for 4 h were exposure to DXM and SA-NPs at the equal DXM for 12 h, respectively. Then, MTT solution (5.0 mg/mL) was added and further incubated for 4 h. After that, the culture medium was discarded and replaced with 200 µL DMSO to dissolve the purple formazan. After shaken for 30 min, the absorbance at 570 nm was determined using a microplate reader (Bio-Rad, model 680, USA), and viability was expressed as the percentage of the control. All of experiments were repeated thrice.

### Renal IRI induction and treatment protocol

ICR male mice (Zhejiang Medical Animal Centre, Hangzhou, China) was used in this study. Age- and weight-matched mice were anesthetized with an intraperitoneal injection of pentobarbital sodium (1%, 50 mg/kg). The renal pedicle was exposed using a dorsal lumbotomy incision, and the renal arteries were subjected to bilateral clamping for 30 min at room temperature, followed by reperfusion, which was ensured by visual inspection of the kidneys (Kumar et al., 2009). Sham-operated animals had an incision plus 30 min of waiting time without clamping. After ischemia or sham surgery, flank muscle and skin layers were sutured, and 1 ml of pre-warmed 0.9% saline solution was subcutaneously administered immediately before closing the incision to prevent dehydration.

Mice were randomly allocated into the following groups: (1) Sham + saline group (*n* = 6); (2) IRI + saline group (*n* = 6); (3) IRI + DXM (*n* = 6); (4) IRI + NPs (*n* = 6); (5) IRI + SA-NPs (*n* = 6). At 24 h after intravenous administration, mice were killed, and blood samples and kidneys were collected for measurements.

### Tissue distribution of SA-NPs

Near infrared dye indocyanine green (ICG) was used to label SA-NPs (SA-NPs-ICG) as following: 1 mg SA-PEG-DXM, 7.7 mg GM, 1 mg OA and 0.3 mg ICG were dissolved in 1 mL ethanol and rapidly dispersed into 10 mL deionized water under mechanical stirring with 400 rpm at 60 °C for 10 min. Then, SA-NPs-FITC was collected by centrifugation at 20,000 rpm for 15 min, and subjected to further use. The preparation of NPs-ICG followed the identical procedures as SA-NPs-ICG.

RETRACTED

IRI mice were injected intravenously with SA-NPs-ICG or NPs-ICG at the same dose of ICG. The mice were sacrificed at predetermined times (1, 2, 4, 6, 12 and 24 h) and organs were harvested, including the heart, liver, spleen, lung, and kidney. Fluorescence signal in collected tissues was analyzed using the Maestro in vivo imaging system (Cambridge Research & Instrumentation, Inc., Woburn, MA, USA).

Then, DXM distribution in IRI mice were quantificationally investigated using ultra performance liquid chromatography (UPLC) method. Mice were randomized into three groups (*n* = 3) and injected intravenously with DXM, NPs and SA-NPs at a dosage of 1.2 mg DXM/kg body weight, respectively. At predetermined times (6 and 12 h), mice were sacrificed by cervical dislocation and tissue samples were harvested, including the heart, liver, spleen, lung, and kidney. After washed with saline, the samples were homogenized and extracted with ethyl acetate, and then vortexed for 5 min and centrifugated for 10 min at 3000 r/min. The supernatants were collected and evaporated to dryness. The obtained dry residues were dissolved in methanol and filtered through a 0.22 µm syringe filter. The filtrate was collected for UPLC analysis. Tissue distribution was expressed as the amount of DXM per gram of the tissues (Xiang et al., 2007).

### Biochemical analysis

Renal function was assessed via determining serum creatinine (Scr) and blood urea nitrogen (BUN). Serum samples were determined using an automated Beckman Analyzer (Beckman Instruments GmbH, Munich, Germany). All of experiments were repeated thrice.

### Histological examination

Renal tissues were fixed in 4.5% buffered formalin and embedded in paraffin. The sections were stained with hematoxylin and eosin (H&E) for morphology analysis using a fluorescence microscope (Olympus, Japan). Examination was carried out in a blinded fashion by an experienced pathologist. The following parameters were used to assess renal morphological damages: epithelial necrosis, luminal necrotic debris, and tubular dilation (Nlandu-Khodo et al., 2016).

### Detection of pro-inflammatory cytokines and oxidative stress

The levels of TNF-α, interleukin-6 (IL-6) were determined using ELISA kits according to the manufacturer’s protocols (Boster Co., Ltd., Wuhan, China). The levels of superoxide dismutase (SOD), malondialdehyde (MDA), glutathione (GSH) and myeloperoxidase (MPO) were measured using commercial kits according to the manufacturer’s protocols (Nanjing Jiancheng Bioengineering Institute, Nanjing, China). All of experiments were repeated thrice.

### TUNEL assay

In the *in vivo* model, a terminal deoxynucleotidyl transferase-mediated dUTP nick-end labeling (TUNEL) assay (Milipore, MA, USA) was used to detect apoptotic cells according to the manufacturer’s protocol. The mount of apoptosis cells were counted at ×400 magnification and 10 fields per slide for each samples were randomly selected. For the *in vitro* experiment (Han et al., 2012), apoptotic cells were detected via TUNEL staining and then labeled with Hoechst 33258 to determine the amount of total nuclei. Fluorescence micrographs were taken using a fluorescence microscope (Olympus, Japan). TUNEL positive cell rate (%) was calculated as the following formula:

$$TUNEL\;positive\;cell\;rate\;(\%)\;=\;\frac{The\;number\;of\;TUNEL-positive\;nuclei}{The\;number\;of\;total\;nuclei}\;\times \;100\%$$

RETRACTED

### Immunofluorescent and immunohistochemical staining

All staining of kidney were performed on 4 µm paraffin sections as previously described. Briefly, cryosections were air-dried and then primary antibody against Kidney injury molecule-1 protein (Kim-1, 1:200, proteintech). The slides were exposed to Cy3-labeled (1: 500) secondary antibody (Cell Signaling Technology, USA) and captured with fluorescence microscope (Olympus, Japan). Immunohistochemical (IHC) staining was performed on formalin-fixed, paraffin-embedded 4 µm sections. E-selectin expression was detected using antibody for E-selectin (dilution of 1:100), and the biotinylated secondary antibody was then added, followed by dimethylaminoazobenzene (DAB) staining. The IHC sections were examined at least 3 times and representative images were presented.

### Western blot

Cells or kidney tissues were homogenized and lysed in ice-cold-modified RIPA lysis buffer. Then, the protein concentrations were determined by a bicinchoninic acid assay (Beyotime Biotechnology, Shanghai, China) according to the manufacturer’s protocol. Samples were matched for protein, separated by SDS–PAGE, and transferred to PVDF membranes (Sigma-Aldrich). After blocked at room temperature for at least 1 h in blocking buffer, the membranes were blotted with anti-Bax (1:2000, Abcam), anti-Bcl (1:2000, Abcam), anti-Caspase 3 (1:2000, Abcam), anti-Caspase-9 (1:2000, proteintech), anti-CD62E (E-selectin, 1:2000, Abcam) and anti-β-actin (1:2000, proteintech) antibodies overnight at 4 °C. The blots were washed and incubated with the secondary ant-rabbit immunoglobulin G (IgG) horseradish peroxidase (HRP) (1:3000, Beyotime Biotechnology, Shanghai, China) for 1 h at room temperature. The membrane was exposed to Fuji Medical X-ray film (Fujifilm) for various periods in a film cassette. The target bonds were selected and the average density was calculated. To facilitate comparisons, densitometry values of target protein were standardized with that of β-actin (Son et al., 2017).

RETRACTED

### Adverse effects during DXM therapy

Given glucocorticoids potentially lead to lymphocytopenia (Czock et al., 2005), lymphocyte count was detected after SA-NPs treatment once every 3 days on day 0, 3, 6, 9, 12 and 15 (the initial administration was set as day 0). Lymphocytes were counted in blood sampled from orbits.

The effect of DXM on bone mineral density (BMD) was also investigated in this study because long-term treatment with glucocorticoids causes osteoporosis by various mechanisms affecting osteoblastic and osteoclastic functions (Schacke et al., 2002; Engelbrecht et al., 2003). Mice were weighed every three days, and doses were adjusted according to the body weight. Mice were injected intravenously with DXM and SA-NPs (*n* = 3) once every 3 days on day 0, 3, 6, 9 and 12. On the 15th day, femur were harvested and determined by dual energy X-ray absorptiometry (XR-36, NORLAND, USA).

### Statistical analysis

All values are reported as mean ± standard deviation (SD) unless otherwise stated. All statistical analysis was performed using SPSS 14.0 statistical software. The significant differences between the groups were analyzed by a Student’s t test. Comparisons among multiple groups were analyzed by one-way analysis of variance (ANOVA). Data were considered statistically to be significant at *p* < .05.

## Results and discussion

### Preparation and characterization of SA-NPs

SA-PEG-DXM was first synthesized according to our previous report (Hu et al., 2017). The synthesis illustration of SA-PEG-DXM is shown in Figure S1. The chemical structures of SA-PEG-DXM were confirmed by proton spectra and provided in Figure S2. SA-NPs containing different OA contents were prepared via solvent diffusion method in an aqueous system and characteristics, such as size, DPI, zeta potential, encapsulation efficiency (%) and drug content (%), were provided in Table 1, NPs as control. The mean diameters of SA-NPs and NPs were 35.6 ± 5.9 nm and 40.1 ± 9.5 nm, respectively. The TEM images showed that SA-NPs and NPs were both spherical with smooth surfaces (Figure 1(A)). The particle sizes of discrete spheres were consistent with hydrodynamic diameter estimated from DLS analysis. Zeta potential is a key value indicating the stability of colloidal dispersion. As shown in Table 1, the absolute value of zeta potential of SA-NPs and NPs were both above 30 mV (−34.3 ± 1.1 mV *versus* − 31.2 ± 0.5 mV, SA-NPs *versus* NPs). The high negative zeta potential contributes to prevent the particle aggregation and then enhance the stability of particles via electrostatic repulsion (Wei & Ge, 2012). The encapsulation efficiency and drug content of SA-NPs were 94.08 ± 0.3% and 2.82 ± 0.09%, respectively. The amount of DXM in SA-NPs included two sections, encapsulated DXM and conjugated DXM in SA-PEG-DXM. Although the proportion of encapsulated DXM and conjugated DXM could not be confirmed in this study, it had no effects on the follow-up experiments. Figure 1(B,C) showed that size and PDI of SA-NPs were nearly unchanged over 4 days at 37 °C, indicating SA-NPs potentially had good colloidal stability in human body (Wang et al., 2016).

RETRACTED

**Figure 1.** Characterization of SA-NPs. (A) The size distribution obtained by DLS and TEM images of NPs and SA-NPs. (B) and (C) *In vitro* stability of SA-NPs at 37 °C in pH 7.4 PBS, including size and PDI. Data were presented as mean ± SD (*n* = 5). (D) The DXM release behaviors of NPs and SA-NPs at 37 °C in pH 7.4 PBS. Data were presented as mean ± SD (*n* = 3).

**Table 1.** Characterization of NPs and SA-NPs (*n* = 3).

Groups	Size(nm)	PDI	Zeta	EE(%)	DC(%)
SA-NPs (10% OA)	35.6 ± 5.9	0.242 ± 0.021	−34.3 ± 1.1	94.08 ± 0.3	2.82 ± 0.09
NPs (10% OA)	40.1 ± 9.5	0.237 ± 0.023	−31.2 ± 0.5	93.20 ± 0.6	2.80 ± 0.12

PDI: polydispersity index; EE: encapsulation efficiency; DC: drug content.

### *In vitro* drug release behavior of SA-NPs

The *in vitro* drug release behavior of SA-NPs was studied via the dialysis method and the results were shown in Figure 1(D). Free DXM released rapidly, more than 90% within 12 h. In contrast, DXM release from SA-NPs could be maintained for more than 48 h, suggesting SA-NPs showed relatively low leakage at 37 °C and pH 7.4. In addition, NPs showed similar release behavior with SA-NPs, indicating SA had no effects on the release behavior of SA-NPs. The released DXM from SA-NPs also included two sections, encapsulated DXM and conjugated DXM in SA-PEG-DXM. The conjugated DXM from SA-PEG-DXM was due to the hydrolysis of ester bond, and its release behavior within 48 h was provided in Figure S3.

### Cellular uptake of SA-NPs

The cellular uptake of SA-NPs by HUVECs was investigated by labeling SA-NPs with FITC and visualizing the internalization of SA-NPs using a fluorescence microscope. As shown in Figure 2(A), the FITC fluorescent intensity of the H_2_O_2_-pretreated cells incubated with SA-NPs-FITC was stronger than that of cells incubated with NPs-FITC in a time-dependent manner. Its fluorescent intensity was also higher than those of cells without H_2_O_2_-pretreatment incubated with SA-NPs-FITC and NPs-FITC. Flow cytometry was further used to quantitatively investigate the internalization behaviors of SA-NPs. As shown in Figure 2(B), a 1.75-, 1.6- and 1.5-fold increase in the internalization of SA-NPs-FITC by H_2_O_2_-pretreated cells was in comparison to NPs-FITC internalized by H_2_O_2_-pretreated cells after 1, 2 and 6 h incubation, respectively (*p < .05). Moreover, no significant difference was observed in the cellular uptake of SA-NPs-FITC and NPs-FITC by cells without H_2_O_2_-pretreatment. The increased cellular uptake of SA-NPs-FITC by H_2_O_2_-pretreated HUVECs may result from the affinity of SA to E-selectin receptor.

RETRACTED

**Figure 2.** The enhanced cellular internalization of SA-NPs *in vitro*. (A) The fluorescent images of HUVECs with or without H_2_O_2_-pretreatment at different post-exposure time to NPs-FITC and SA-NPs-FITC, respectively. The scale bar =100 μm. (B) Flow cytometry results of internalization behaviors of SA-NPs by H_2_O_2_-pretreated HUVECs after 1, 2 and 6 h incubation, respectively. Data were presented as mean ± SD (*n* = 3), *p < .05. (C) The fluorescent images of HUVECs with H_2_O_2_-pretreatment at 2 h post-exposure to SA-NPs-FITC. The scale bar =60 μm. (D) Semi-quantitative results of fluorescent images of (c). (E) Intracellular fluorescence intensity determined by flow cytometry during HUVECs with various concentrations of SA at 2 h post-exposure to SA-NPs-FITC.

To testify the enhanced cellular uptake of SA-NPs was associated with the specific binding of SA to E-selectin receptor expressed on H_2_O_2_-pretreated HUVECs, cells with and without H_2_O_2_-pretreatment were incubated with SA-NPs-FITC for 2 h, respectively. As shown in Figure 2(C,D), the fluorescence intensity of SA-NPs-FITC in H_2_O_2_-pretreated cells was much stronger than that in cells without H_2_O_2_-pretreatment. Meanwhile, the expression of E-selectin receptor in cells with H_2_O_2_-pretreatment was higher than that in cells without H_2_O_2_-pretreatment, which was consistent with the difference of fluorescence intensity of SA-NPs-FITC, indicating the predominant endocytosis was mediated by E-selectin receptor. Competitive assay was performed to further testify this E-selectin receptor-involved internalization process using flow cytometry. As shown in Figure 2(E), free SA could significantly reduce the uptake of SA-NPs-FITC in a dose-dependent manner (0.5, 1.0 and 2.0 mg/mL). The results demonstrated E-selectin receptor-mediated internalization of SA-NPs, and SA in SA-NPs played a key role during this process.

### SA-NPs protect HUVECs against oxidative stress damage

To investigate whether SA-NPs protected HUVECs against oxidative stress damage, a MTT assay was used to assess cell viability. Cell survival was investigated after DXM, NPs, and SA-NPs treatment in HUVECs pretreated with H_2_O_2_. Firstly, cell survival of HUVECs incubated with a range of concentrations of H_2_O_2_ (from 100 µmol/L to 800 µmol/L) was investigated and the results showed that H_2_O_2_ decreased cell survival in a dose-dependent manner (Figure S4). To present a maximum dynamic range for assessing protective vs. harmful responses, 200 µmol/L H_2_O_2_ incubation of 4 h was used in the following assays. As shown in Figure 3(A), cell survival of HUVECs at 4 h post-exposure to 200 µmol/L H_2_O_2_ decreased sharply, whereas both DXM and SA-NPs (DXM 10 µmol/L, both *p < .05) reduced H_2_O_2_-dependent damage and restored cell survival following the oxidative stress.

RETRACTED

**Figure 3.** SA-NPs protect HUVECs against oxidative stress damage. (A) SA-NPs ameliorate cell survival of HUVECs pretreated with 200 µmol/L H_2_O_2_, and cell viability was determined by MTT assay. (B) The fluorescent images of 200 µmol/L H_2_O_2_-pretreated HUVECs treated with SA-NPs and then subjected to TUNEL staining. The scale bar =100 μm. (C) The number of TUNEL-positive nuclei was expressed as a percentage of total nuclei detected by Hoechst staining. (D) Representative western blot analysis of Bax, Bcl-xL, Caspase-3 and Caspase-9 in 200 µmol/L H_2_O_2_-pretreated HUVECs treated with DXM and SA-NPs, β-actin was used as control. (E) Densitometric analysis for detecting the levels of Bax. (F) Densitometric analysis for detecting the levels of Bcl-Xl. (G) Densitometric analysis for detecting the levels of Caspase-3. (H) Densitometric analysis for detecting the levels of Caspase-9. Values were normalized against β-actin. Data were presented as mean ± SD (*n* = 3), *p < .05.

Based on the TUNEL and Hoechst 33258 staining, H_2_O_2_-pretreated HUVECs showed the decreased cell viability, as reflected by the high level of TUNEL-positive staining. After exposure to DXM and SA-NPs (DXM 10 µmol/L), the declined TUNEL-positive rates were observed in Figure 3(B,C), indicating SA-NPs protected HUVECs against H_2_O_2_-induced apoptosis. Apoptosis-related proteins, including Bax, Bcl-xL, Caspase-3 and Caspase-9 (Singh et al., 2013), were examined using western blot analysis to confirm whether H_2_O_2_-induced cell death was associated with apoptosis. As shown in Figure 3(D–G), the abnormal changes in the expression of Bax, Bcl-xL, Caspase-3 and Caspase-9 were normalized after treatment with DXM and SA-NPs, respectively (*p < .05).

### Distribution of SA-NPs

The expression of E-selectin receptor in the kidneys from IRI-induced AKI mice was investigated using immunohistochemical staining. As shown in Figure 4(A), the expression of E-selectin receptor in IRI group (black arrow) was higher than that from sham group. Immunoblotting also revealed the increased E-selectin in IRI group in comparison to sham group (Figure 4(B,C), *p < .05). The renal overexpression of E-selectin receptor in IRI mice provided the reasonable basis for the renal-targeting therapy of SA-NPs.

RETRACTED

**Figure 4.** Renal-targeting efficacy of SA-NPs. (A) Representative immunological histological chemistry images of E-selectin in kidney sections, including sham and IRI mice. Positive expression was labeled with black arrow. (B) Representative western blot analysis of E-selectin protein expression in kidneys from sham and IRI mice. (C) Densitometric analysis for detecting the levels of E-selectin. Data were presented as mean ± SD (*n* = 3), *p < .05. (D) The fluorescence signal image of excised major organs (heart, liver, spleen, lung, and kidney) in IRI mice treated with ICG-labeled NPs and SA-NPs at 6 h postinjection. (E) The renal fluorescence signal image of IRI mice treated with ICG-labeled NPs and SA-NPs for various point-in-times. (F) The tissue distribution of DXM, NPs and SA-NPs in IRI mice at 6 and 12 h after intravenous administration at a dose of 1.2 mg/kg DXM, respectively. Data were presented as mean ± SD (*n* = 3), *p < .05.

Near infrared dye ICG was used to label SA-NPs (SA-NPs-ICG) to investigate the kidney-targeting efficacy in IRI mice, ICG-labeled NPs (NPs-ICG) as control. As shown in Figure 4(D), the higher renal fluorescence signal in mouse treated with SA-NPs-ICG at 6 h postinjection was observed in comparison to that treated with NPs-ICG, suggesting the increased accumulation of SA-NPs-ICG in renal tissue due to the specific interaction between SA of SA-NPs-ICG and E-selectin receptor on vascular endothelial cells. Then, the renal accumulation of SA-NPs-ICG and NPs-ICG in IRI mice at different point-in-time (1, 2, 4, 6, 12, and 24 h) was investigated and the results were shown in Figure 4(E). The renal fluorescence signal of SA-NPs-ICG could be maintained for more than 24 h and reached the maximum at 6 h after intravenous administration. In contrast, the renal fluorescence signal of NPs-ICG was lower than that of SA-NPs-ICG at each point-in-time.

The renal-targeting ability of SA-NPs was further investigated via determining DXM content in major organs using UPLC assay. IRI mice were respectively treated with DXM, NPs, and SA-NPs at 1.2 mg/kg equivalent DXM and the results were shown in Figure 4(F). After administration for 6 and 12 h, the accumulation of SA-NPs in renal tissue was significantly enhanced in comparison to DXM and NPs (both *p < .05). Especially at 6 h, the renal DXM contents in IRI mice treated with SA-NPs were 2.7- and 5.88-fold higher than those treated with DXM and NPs, respectively. Although the accumulation of SA-NPs in liver was inevitably increased, no abnormal liver function indexes and histological changes were detected (Figure S5 and S6). Bio-distribution experiments in IRI mice suggested SA-NPs had significant renal specificity, which was associated with the following reasons that SA-NPs could be recognized by E-selectin receptor expressed on vascular endothelial cells during IRI, and then internalized into cells.

RETRACTED

### Renal functions in IRI mice after SA-NPs therapy

Renal function indexes, including Scr and BUN, were used to assess the therapeutic outcomes in DXM-treated IRI mice, and the results were shown in Figure 5(A,B). Compared with sham group, IRI group caused significant renal dysfunction at 24 h as suggested by significant increase in Scr (0.528 ± 0.035 *versus* 0.313 ± 0.012 mg/dl; IRI *versus* sham, *p < .05) and BUN (74.1 ± 5.3 *versus* 18.5 ± 3.2 mg/dl; IRI *versus* Sham, *p < .05). After treated with SA-NPs, both Scr (0.528 ± 0.035 *versus* 0.362 ± 0.031 mg/dl; IRI *versus* IRI + SA-NPs, *p < .05) and BUN (74.123 ± 5.251 *versus* 29.467 ± 6.376 mg/dl; IRI *versus* IRI + SA-NPs, *p < .05) were significantly improved in comparison to IRI group. Moreover, SA-NPs treatment showed the better therapeutic outcomes than DXM and NPs treatments, as showed in Scr (0.426 ± 0.016 *versus* 0.362 ± 0.031 mg/dl, IRI + DXM *versus* IRI + SA-NPs, *p < .05; 0.456 ± 0.021 *versus* 0.362 ± 0.031 mg/dl, IRI + NPs *versus* IRI + SA-NPs, *p < .05) and BUN (42.367 ± 6.981 *versus* 18.501 ± 3.161 mg/dl, IRI + DXM *versus* IRI + SA-NPs, *p < .05; 64.067 ± 5.515 *versus* 18.501 ± 3.161 mg/dl, IRI + NPs *versus* IRI + SA-NPs, *p < .05). The different therapeutic outcomes between DXM and NPs responded to the discrepant DXM content in kidneys (6.274 ± 1.258 *versus* 2.883 ± 1.120 µg/g, DXM *versus* NPs, *p < .05; Figure 4(F)), which was potentially associated with the following reasons: 1) The prolonged release of DXM from NPs led to the lower drug concentration in comparison to free DXM. 2) Compared with free DXM, the increased accumulation of NPs in liver because NPs were liable to retention by reticuloendothelial system (RES).

**Figure 5.** SA-NPs ameliorate renal functions in IRI mice. (A) The abnormal increase of Scr in renal IRI mice was abrogated by SA-NPs. (B) The abnormal increase of BUN in renal IRI mice was abrogated by SA-NPs. Data were presented as mean ± SD (*n* = 3), *p < .05. (C) Representative H&E staining images of kidney sections. The scale bar = 100 μm. (D) Light photomicrographs of renal TUNEL staining results in IRI mice after SA-NPs therapy. The scale bar = 100 μm. (E) TUNEL-positive rates of renal sections in IRI mice after SA-NPs therapy. Data were presented as mean ± SD (*n* = 3), *p < .05.

RETRACTED

### Histopathology of kidneys from IRI mice after SA-NPs therapy

Kidneys from IRI mice were analyzed by H&E staining after SA-NPs therapy, DXM and NPs as control. Histopathologic images (Figure 5(C)) indicated the kidneys from IRI mice had the widely spread cellular infiltration and remarkable tubular lumen dilatation. In addition, degeneration and necrosis of the renal tubular epithelial cells could also be observed in focal areas. These focal changes were distributed in the whole kidney cortex. Compared with IRI group, the renal damage was ameliorated at a certain extent after DXM and NPs treatment, though dilatation of the tubular lumen and luminal congestion could still be found. In contrast, SA-NPs group showed mild degeneration of the renal tubular cells and dilatation of the tubular lumen at the same time point.

Apoptosis is a major pathological process in kidney injury, and it can be triggered by infiltration of inflammatory cells and oxidative stress (Pressly et al., 2017). *In vitro* assay has demonstrated the anti-apoptosis of SA-NPs. Apoptosis of renal cells *in situ* was then examined and the results were shown in Figure 5(D,F). Renal section from IRI mice showed extensive nuclear changes in line with apoptotic cell death, with apoptotic index (AI) = 81.4 ± 8.3% (IRI *versus* sham, *p < .05). In contrast, few TUNEL-positive cells were observed in renal sections from sham group (AI =6.5 ± 2.8%). Evident decline in AI was observed in IRI mice after DXM and NPs therapy (AI =48.8 ± 4.2% and AI =76.3 ± 4.5%), and the further reduction in AI was found in mice treated with SA-NPs (AI =37.2 ± 3.9%, IRI + SA-NPs *versus* IRI + DXM, IRI + SA-NPs *versus* IRI + NPs, *p < .05).

### Changes of oxidative stress levels and pro-inflammatory cytokines in IRI mice after SA-NPs therapy

To confirm the protective mechanisms of SA-NPs *in vivo*, the levels of oxidative stress in IRI mice were assessed. As shown in Figure 6(A,B), the levels of SOD and GSH were significantly reduced in IRI mice (IRI *versus* Sham, *p < .05). The SOD and GSH levels in IRI mice were improved after DXM, NPs, and SA-NPs therapy, respectively. Moreover, SA-NPs therapy showed the better therapeutic outcomes than DXM and NPs (IRI + SA-NPs *versus* IRI + DXM, IRI + SA-NPs *versus* IRI + NPs, both *p < .05). Compared with sham mice, MDA level was higher in IRI mice (IRI *versus* Sham, *p < .05; Figure 6(C)). After treatment with DXM-based formulations, MDA levels were enhanced and SA-NPs therapy showed the better therapeutic effect than DXM and NPs (IRI + SA-NPs *versus* IRI + DXM, IRI + SA-NPs *versus* IRI + NPs, both *p < .05).

RETRACTED

**Figure 6.** Changes of oxidative stress and pro-inflammatory cytokines in IRI mice after SA-NPs therapy. (A), (B) and (C) SA-NPs exerted anti-oxidative effects against renal IRI, and the levels of SOD, GSH, and MDA were determined in IRI mice after SA-NPs therapy. (D) Renal MPO activity was determined in IRI mice after SA-NPs therapy. (E) and (F) The levels of cytokines (TNF-α and IL-6) were determined in IRI mice after SA-NPs therapy. Data were presented as mean ± SD (*n* = 3), *p < .05.

MPO was also determined to assess leukocyte infiltration, and the results were shown in Figure 6(D). MPO level was significantly increased in IRI mice, which was inhibited by the DXM-based formulations, and SA-NPs therapy showed the better therapeutic outcomes than DXM and NPs (IRI + SA-NPs *versus* IRI + DXM, IRI + SA-NPs *versus* IRI + NPs, both *p < .05). To further show the inflammatory states, pro-inflammatory factors, including TNF-α and IL-6, were checked in this study. As shown in Figure 6(E,F), cytokine levels in IRI mice were sharply increased (TNF-α, 8.53 ± 0.70 *versus* 2.63 ± 0.35 ng/mg protein, IRI *versus* sham, *p < .05; IL-6, 6.52 ± 0.51 *versus* 1.52 ± 0.21 pg/mg protein, IRI *versus* sham, *p < .05). After treatment with DXM-based formulations, the abnormal TNF-α and IL-6 levels were improved, and SA-NPs therapy showed the better anti-inflammatory effects than DXM and NPs (IRI + SA-NPs *versus* IRI + DXM, IRI + SA-NPs *versus* IRI + NPs, both *p < .05).

### Safety assessment

Adverse effects after SA-NPs therapy were also examined in this study. Long-term and systematic administration of DXM is always accompanied by several drug-induced side effects, such as abnormal lymphocyte count and osteoporosis. As shown in Figure 7(A), free DXM would lead to the reduced lymphocyte count. In contrast, the lymphocyte count was normalized in IRI mice treated with SA-NPs (SA-NPs *versus* DXM, *p < .05), which was associated with the lower accumulation of SA-NPs in lymphoid organs.

**Figure 7.** The reduced adverse effects of SA-NPs in IRI mice. (A) The improved lymphocyte count in IRI mice after SA-NPs therapy. (B) The improved bone mineral density in IRI mice after SA-NPs therapy. Data represent mean ± SD (*n* = 3), *p < .05.

Then, BMD was determined by dual energy X-ray absorptiometry to assess whether SA-NPs could alleviate the osteopenic effect resulted from DXM. Previous studies have demonstrated DXM, one of glucocorticoid agents, might reduce BMD along with the defective osteoblastogenesis and osteoclastogenesis in the bone marrow and apoptosis of mature osteoblasts and osteocytes (Komori, 2016). Determination of BMD is a good way for early diagnosis of osteoporotic disease and it was hence used as an index in this study. As shown in Figure 7(B), the reduced DXM induced by DXM was improved with SA-NPs therapy in comparison to free DXM (0.089 ± 0.007 g/cm^2^ *versus* 0.106 ± 0.007 g/cm^2^, IRI + DXM *versus* IRI + SA-NPs, *p < .05). Hence, it was reasonable to demonstrate that SA-NPs could reduce the extrarenal response of DXM.

RETRACTED

## Conclusions

Ischemia-reperfusion-induced kidney injury is an inevitable consequence of kidney transplantation. It causes a serious inflammatory response associated with the generation of reactive oxygen species, endothelial dysfunction, and induction of pro-inflammatory molecules. Therefore, anti-oxidative stress therapy is of great importance for post renal IRI. Based on our experimental studies, we demonstrated that SA-modified solid lipid NPs could be used as a promising drug delivery system for ischemia-reperfusion-induced acute renal injury via specific recognition by E-selectin receptor expressed on vascular endothelial cells.

## Supplementary Material

IDRD_Du_et_al_Supplemetal_Content.docx
